The article "Comparison of Efficacy and Safety of Different Doses of Dexmedetomidine for Epidural Labor Analgesia" was published in 2023. Journal: Emerg Med Int.

# Comparison of Efficacy and Safety of Different Doses of Dexmedetomidine for Epidural Labor Analgesia

**DOI:** 10.1155/2023/2358888

**Published:** 2023-04-04

**Authors:** Liang Ge, Peng Zhang, Lingguo Kong, Wei Wang, Qian Tong, Quanlong Fan, Xudong Han

**Affiliations:** ^1^Department of Anesthesiology, Gansu Provincial Maternity and Child-Care Hospital (Gansu Provincial Central Hospital), Lanzhou, Gansu 730050, China; ^2^The Reproductive Medicine Special Hospital of the 1st Hospital of Lanzhou University, Lanzhou, Gansu 730000, China; ^3^Key Laboratory for Reproductive Medicine and Embryo, Lanzhou, Gansu 730000, China

## Abstract

**Objective:**

To explore the efficacy and safety of different doses of dexmedetomidine (DEX) for epidural labor analgesia (ELA).

**Methods:**

From June 2021 to June 2022, 147 parturients who underwent ELA in our hospital were selected and divided into low- (0.5 *μ*g/kg DEX), medium- (0.75 *μ*g/kg DEX), and high-dose (1.0 *μ*g/kg DEX) groups (*n* = 49 for each) according to the random number table method. The analgesic effect was assessed using the Ramsay sedation score and Visual Analogue Scale (VAS), and the labor duration, mean arterial pressure (MAP), and heart rate (HR) before and after analgesia, vaginal bleeding within 2 h postpartum, and delivery outcomes (the cesarean section conversion rate and the neonatal Apgar score) were statistically analyzed. Furthermore, the incidence of adverse reactions was calculated, and maternal satisfaction with delivery was investigated.

**Results:**

After analgesia, the the Ramsay and labor duration were higher in the high-dose group than those in the low- and medium-dose groups, and the VAS scores was lowerin the high-dose group than those in the low- and medium-dose groups(*P* < 0.05), while no difference was identified among the three groups in terms of the cesarean section conversion rate and the neonatal Apgar score (*P* > 0.05). The high-dose group had the greatest fluctuations in MAP and HR levels before and after analgesia than the other two groups, with a higher incidence of adverse reactions (*P* < 0.05). Finally, the survey of delivery satisfaction showed no significant difference in delivery satisfaction among the three groups (*P* > 0.05).

**Conclusion:**

DEX has excellent performance in ELA, which can effectively relieve the pain of puerperae and shorten the labor process. Among them, low-dose DEX has higher safety and is recommended as the first choice. *Trial Registrations*. This trial is registered with ML2021073.

## 1. Introduction

Labor pain is caused by the fact that the fetus passes through the narrow uterus and vagina in the process of natural delivery, and the paroxysmal contractions and friction during fetal movement stimulate the nerve endings of the parturient to generate nerve impulses, which are transmitted to the human brain sensory center along the lumbosacral plexus [1]. Labor pain, as the inevitable product of childbirth, not only brings about physiological pain but also has a great negative impact on the psychology of parturients [2]. In addition to affecting the success rate of delivery, it can also cause maternal psychological diseases such as postpartum depression, which threatens postpartum life [3]. Although cesarean section (CS) can reduce the pain of the parturient during delivery compared with natural childbirth, the traumatic operation may cause greater mechanical damage and other stress reactions [4]. Moreover, because the fetus directly contacts the outside without being squeezed by the birth canal, its innate immunity is low, and it is more at risk of various postpartum diseases than the fetus in natural childbirth [5].

Therefore, the management of labor pain greatly determines the final outcome of childbirth. At present, epidural analgesia is the first choice for clinical labor analgesia; it achieves better analgesic effects through local anesthesia, which not only allows mothers to participate in the whole labor process consciously but is also more convenient for doctors to operate and can reduce the proportion of CS; meanwhile, local anesthesia will cause no motor block nor uterine inertia [6, 7]. Among the anesthetic drugs, dexmedetomidine (DEX), as an agonist of *α*_2_ receptor, is often used in combination with other agents in clinical epidural anesthesia, with the effects of prolonging the effectiveness of local anesthetics, reducing the dosage of anesthetic drugs, and alleviating pain [8]. It has been reported [9] that 0.1% ropivacaine combined with 0.25, 0.5, 0.75, and 1.0 *μ*g/mL DEX continuous epidural infusion is used for labor analgesia, and the results show that different doses of DEX have different analgesic effects. However, it is still controversial whether lower drug dosages can achieve the ideal labor analgesic effect.

Accordingly, to confirm the optimal dosage of DEX in epidural labor analgesia (ELA), this study used different doses of DEX for analgesic treatment of laboring mothers so as to provide a more reliable medication reference for future clinical selection of labor analgesia and ensure the life safety of mothers and newborns.

## 2. Data Acquisition

The sample size of this study was estimated based on the sample content estimation formula of multiple sample mean comparisons of the grouped design data as follows:

(1) $$\begin{array}{c} n=\frac{\varphi^{2}\left(\sum_{i=1}^{k}\sigma_{i}^{2}/k\right)}{\left(\sum_{i=1}^{k}{\left(\mu_{i}-\mu \right)}^{2}/\left(k-1\right)\right)}\text{,} \end{array}$$

where *μi* was the overall mean of each group and was replaced by the mRNA mean of each group obtained in the preliminary investigation, which was 2.55 (low-dose group), 2.23 (medium-dose group), and 2.71 (high-dose group), respectively; Σ*i* was the population standard deviation of each group and was replaced by the standard deviation of mRNA obtained in the preliminary investigation of each group, which was 1.08 (low-dose group), 1.04 (medium-dose group), and 1.21 (high-dose group), respectively; and *K* is the number of sample groups, equal to 3. The test level *α* = 0.05, test efficiency 1 − *β* = 0.95, *νi* = k − 1 = 2, *ν*_2_ = ∞, and the lookup table obtained Φ = 2.52. Substituting into the above formula, we calculated the required sample size of *n* ≈ 44 cases in each group. After considering the loss of a follow-up rate of 10%, a total of 49 patients were included in each group, and finally, 147 cases were included in this study.

One hundred and forty-seven parturients undergoing ELA in our hospital from June 2021 to June 2022 were selected and randomly divided into low-, medium-, and high-dose groups, each with 49 cases. Ethical approval was obtained from the hospital's ethics committee, and informed consent was obtained from each participant.

### 2.1. Eligibility Criteria

The criteria for patient enrollment were as follows: (1) age 20–35, (2) feasibility for vaginal delivery after obstetric evaluation, (3) singleton and full-term pregnancy with fetal presentation, and (4) no pregnancy-related complications (e.g., pregnancy-induced hypertension, gestational diabetes mellitus, and cholestasis of pregnancy). The criteria for patient exclusion were as follows: (1) smoking/alcohol addiction or history of drug use, (2) neuroticism, (3) the times of PCA with an epidural analgesia pump during labor analgesia were more than 3 times, and (4) duration from the onset of labor analgesia to fetal delivery >8 h. The criteria for elimination were as follows: (1) those who did not follow the original treatment plan and used other interventions in the trial, (2) those who requested withdrawal, and (3) those who provided false information.

### 2.2. ELA

ELA started when the mother entered the delivery room with the cervix opened by 2-3 cm. The analgesic drugs used were sufentanil (Yichang Renfu Pharmaceutical Co. Ltd., 50 *μ*g/1 mL) + ropivacaine (AstraZeneca, UK, 75 mg/10 mL). The initial dose of ELA was 0.08% ropivacaine + 0.4 *μ*g/mL sufentanil (10 mL) via an epidural bolus injection, with a background dose of the pulse pump of 10 mL/h and a PCA of 6 mL/h.

### 2.3. DEX Pump Injection

Immediately after labor analgesia, the parturient was pumped with DEX intravenously, with the dose in the low-, medium-, and high-dose groups being 0.5 *μ*g/kg, 0.75 *μ*g/kg, and 1.0 *μ*g/kg, respectively. The anesthetics were all pumped within 10 min.

### 2.4. Scoring Criteria

The sedation degree was evaluated using the Ramsay Sedation Scale [10] at 1 h, 2 h, and 4 h after labor analgesia. The grading criteria were as follows: grade 6: no response to tapping between eyebrow or strong sound stimulation; grade 5: slow response to eyebrow tapping or strong sound stimulation; grade 4: quick response to eyebrow tapping or strong sound stimulation; grade 3: responds to commands only; grade 2:patient cooperation and good orientation; and grade 1: anxiety, restlessness, or irritability. Pain assessment, which was made before analgesia (T0), 1 hour after analgesia (T1), during the first stage of labor with the orifice of the uterus opened by 7-8 cm (T2), and during the second stage of labor with complete opening of the uterus orifice (T3), employed the Visual Analogue Scale (VAS). Out of 10 points, a score of 0–2 indicates that the mother is in a good mood, with a quiet face and quick responses to questions; 3–5 means that the mother is quiet with no agitation and an indifferent face and responds to commands only; 6–8 suggests emotional anxiety or depression in the mother, with a slightly painful face and reluctant responses; and >8 corresponds to a painful face with forced posture and inability to respond. The Apgar score [11] was utilized to assess neonatal status 1 min and 5 min after birth, investigating neonatal activity, pulse, grimace, appearance, and respiration. A score of 10, <7, and <4 suggests normal, mild asphyxia, and severe asphyxia, respectively.

### 2.5. Outcome Measures

(1) The sedative effect was evaluated by the Ramsay score. (2) Pain was assessed by the VAS score. (3) Maternal labor stages were the duration of the first, second, and third stages of labor. (4) Hemodynamics: the maternal mean arterial pressure (MAP) and heart rate (HR) were monitored before, 10 min, and 30 min after analgesia, and vaginal blood loss within 2 h postpartum was recorded. (5) Delivery outcomes were the CS conversion rate and the neonatal Apgar score. (6) Adverse reactions (ARs): the ARs from the beginning of analgesia to the completion of labor were counted, and the incidence of ARs was calculated. (7) Delivery satisfaction: the delivery satisfaction survey was conducted at the time of discharge, and the results were divided into satisfaction, basic satisfaction, and dissatisfaction. Total satisfaction = (satisfaction + basic satisfaction) cases/total cases × 100%.

### 2.6. Statistical Processing

Data were statistically analyzed by using SPSS 22.0. Counting data were recorded as (%), and a chi-square test was performed to identify the presence or absence of significance among groups. Measurement data, recorded as ($\bar{\chi }$ ± *s*), were analyzed by the variance analysis and LSD intragroup test for significant differences among groups. Results with *P* < 0.05 were considered statistically significant.

## 3. Results

### 3.1. Comparison of Clinical Baseline Data

Comparing the clinical baseline data (age, gestational age, residence, exercise habits, etc.) of the three groups, it can be seen that differences are not statistically significant (*P* > 0.05, Table 1), indicating that the three groups are comparable.

### 3.2. Comparison of Analgesic Effects

The Ramsay score was similar in low- and medium-dose groups at 1 h and 2 h after ELA (*P* > 0.05), which was lower than that of the high-dose group (*P* < 0.05), while the Ramsay score at 4 h after analgesia showed no marked difference among the three groups (*P* < 0.05). In all the three groups, the Ramsay score at 4 h after analgesia was higher than that at 1 h and 2 h after analgesia (*P* < 0.05, Figure 1(a)). In addition, there was no difference in VAS scores among the low-, medium- and high-dose groups at T0 (*P* > 0.05), but the VAS scores at T1–T3 were lower than those at T0, and a decrease in the high-dose group was the most significant (*P* < 0.05, Figure 1(b)).

### 3.3. Comparison of Duration of Labor

Comparing the labor duration among the three groups, it can be seen that the low and medium-dose groups had similar duration of the first, second and third stages of labor (*P* > 0.05), which was higher than that of the high-dose group (*P* < 0.05, Figures 2(a)–2(c)).

### 3.4. Comparison of Hemodynamics

There were differences in neither MAP nor HR among the three groups before analgesia (*P* > 0.05). MAP and HR decreased significantly after analgesia, with their levels at 10 min and 30 min after analgesia showing no evident differences between the low- and medium-dose groups (*P* > 0.05), while the MAP and HR at 30 min after analgesia in the high-dose group were lower than those at 10 min after analgesia (*P* < 0.05, Figures 3(a) and 3(b)). In addition, postpartum hemorrhage differed insignificantly among the three groups (*P* > 0.05, Figure 3(c)).

### 3.5. Comparison of Delivery Outcomes

The conversion to CS was found in 3 parturients in the low-dose group, 3 cases in the medium-dose group, and 4 cases in the high-dose group, showing no statistical significance in the CS conversion rate among the three groups (*P* > 0.05, Figure 4(a)). There were not any notable differences in neonatal 1-min and 5-min Apgar scores among the three groups (*P* > 0.05, Figure 4(b)).

### 3.6. Comparison of ARs

The incidence of ARs was 8.16% in the low-dose group and 12.24% in the medium-dose group, showing no evident difference (*P* > 0.05), while the AR rate in the high-dose group was 26.53%, which was higher than that of the other two groups (*P* < 0.05, Table 2).

### 3.7. Comparison of Delivery Satisfaction

The maternal satisfaction rates with delivery in the low-, medium- and high-dose groups were 80%, 80%, and 80%, respectively, without notable differences among them (*P* > 0.05, Table 3).

## 4. Discussion

In clinical practice, natural delivery is still the preferred mode of delivery, so alleviating the pain of natural delivery has always been a hot spot in modern clinical research. Anesthesia and analgesia, the most common way of labor pain intervention clinically, has its analgesic effects repeatedly verified, but the resulting ARs is still the focus of clinical problems [12, 13]. Researchers believe that the safety of narcotic drugs can be improved by reducing the use of doses [14, 15]. However, it is still controversial whether drug dose reduction is associated with compromised analgesic effects. Therefore, this study can provide reliable reference and guidance for future labor analgesia by exploring the analgesic effects of different doses of DEX on ELA.

In this trial, we used 0.5, 0.75, and 1.0 *μ*g/kg DEX for labor analgesia. The results showed higher Ramsay scores in the high-dose group than those in the low- and medium-dose groups after analgesia, as well as markedly lower VAS scores at T1–T3, suggesting best analgesic effects in the high-dose group. DEX, as an *α*_2_ receptor agonist, exerts a sedative effect mainly by acting on the locus coeruleus receptor in brain tissue, which can reduce the body's stress without influencing the respiratory system [16, 17]. Studies have shown that DEX can exert analgesic effects by stimulating nerve cells to release cholate-like substances to expand the pain threshold of the body [18]. Meanwhile, it can enhance the frequency and intensity of myometrial contractions, reduce uterine bleeding, and accelerate labor, making it suitable for labor analgesia [19, 20]. The analgesic effect of DEX has been confirmed in many previous studies [21–23], but the results of this study have once again demonstrated its excellent application potential, whereas the Ramsay and VAS scores of parturients in the low and medium-dose groups also reached an ideal state after anesthesia, with no evident difference in the number of CS conversions among the three groups, indicating that DEX of 0.5 and 0.75 *μ*g/kg can also meet the need of labor analgesia. Furthermore, we observed that the high-dose group had shorter labor duration than the other two groups, which is also related to the effect of DEX on myometrium contractility mentioned above [24]. However, in the comparison of vital signs, we found more significant alterations in MAP and HR before and after anesthesia in the high-dose group than stale indexes in puerperae in the low-dose group, indicating that low-dose DEX has less influence on maternal hemodynamics. Moreover, the high-dose group was observed to have a higher AR rate than the low- and medium-dose groups, which further indicated that low-dose DEX has higher safety in labor analgesia. In previous studies, we also found that the use of low-dose DEX was more safe for knee replacement and myomectomy [25, 26], which can also support our experimental results. Furthermore, there was no difference in Apgar scores among the three groups of newborns, which also indicates that DEX has little influence on newborns and high application values in labor analgesia. Finally, the results of the maternal satisfaction survey on childbirth also identified no significant differences among the three groups, suggesting that DEX has higher applicability in labor analgesia and can improve parturients' delivery experience. Based on the above experimental results, we believe that, although high-dose DEX has better anesthesia and analgesic effects for parturients, its safety is not ideal. In contrast, low-dose DEX contributes to favorable analgesic effects and safety, which is worthy of recommendation.

However, due to the limited experimental conditions, only young subjects with good physical function were included in this study, and some elderly pregnant women developed DEX rejection that might affect the results. Therefore, more cases from different age groups should be included for confirmation. Second, we need to follow up all the subjects for a longer period of time to confirm the potential longer-term impact of DEX on mothers. Finally, in follow-up research, we should determine the advantages of DEX by using other narcotics as controls so as to further confirm the application value of DEX in ELA.

To sum up, DEX has excellent performance in ELA, which can effectively relieve the pain of puerperae and shorten the labor process. Among them, low-dose DEX has higher safety and is recommended as the first choice.

## Figures and Tables

**Figure 1:** Comparison of analgesic effects. (a) Comparison of the Ramsay score. *Note*. Compared with the low-dose group, ^*∗*^*P* < 0.05; compared with the middle-dose group, ^#^*P* < 0.05; vs. 1 h after ELA, ^&^*P* < 0.05; vs. 2 h after ELA, ^@^*P* < 0.05. (b) Comparison of VAS scores. *Note*. Compared with the low-dose group ^*∗*^*P* < 0.05; compared with the middle-dose group, ^#^*P* < 0.05. *Note*. Compared with the low-dose group, ^*∗*^*P* < 0.05; compared with the middle-dose group, ^#^*P* < 0.05; vs. T1, ^&^*P* < 0.05; vs. T2, ^@^*P* < 0.05; vs. T2, ^^^*P* < 0.05.

**Figure 2:** Comparison of duration of labor. (a) Comparison of first stages of labor. (b) Comparison of second stages of labor. (c) Comparison of third stages of labor. *Note*. Compared with the low-dose group, ^*∗*^*P* < 0.05; compared with the middle-dose group, ^#^*P* < 0.05.

**Figure 3:** Comparison of hemodynamics. (a) Comparison of MAP. (b) Comparison of HR. (c) Comparison of vaginal blood loss within 2 h postpartum. *Note*. Compared with the low-dose group, ^*∗*^*P* < 0.05; compared with the middle-dose group, ^#^*P* < 0.05; vs. before analgesia, ^&^*P* < 0.05; vs. 10 min after analgesia, ^@^*P* < 0.05.

**Figure 4:** Comparison of delivery outcomes. (a) Comparison of 1-min Apgar. (b) Comparison of 5-min Apgar.

**Table 1:** Comparison of clinical baseline data.

	*N*	Age	Gestational week (week)	Place of residence urban/rural	Exercise habits yes/no	Sleeping state normal/bad	Dietary preferences bland/heavy taste
Low-dose group	49	26.02 ± 1.90	39.14 ± 3.09	34/15	16/33	29/20	26/23
Medium-dose group	49	26.51 ± 2.36	40.27 ± 3.03	30/19	13/36	24/25	30/19
High-dose group	49	26.82 ± 2.51	39.31 ± 3.36	32/17	12/37	32/17	30/19
*F* or *χ*^2^		1.545	1.818	0.721	0.879	2.734	0.897
*P*		0.217	0.166	0.698	0.644	0.255	0.639

**Table 2:** Comparison of ARs.

	*n*	Lethargy	Nausea and vomiting	Itching	Breathing depression	Hypotension	Incidence of ARs
Low-dose group	49	2 (4.08)	1 (2.04)	1 (2.04)	0 (0.0)	0 (0.0)	8.16%
Medium-dose group	49	3 (6.12)	2 (4.08)	0 (0.0)	0 (0.0)	1 (2.04)	12.24%
High-dose group	49	5 (10.20)	3 (6.12)	2 (4.08)	1 (2.04)	2 (4.08)	26.53%^*∗*^
*χ * ^2^							6.907
*P*							0.032

*Note.* Compared with the low-dose group, ^*∗*^*P* < 0.05.

**Table 3:** Comparison of delivery satisfaction.

	*n*	Satisfaction	Basic satisfaction	Dissatisfaction	Total satisfaction
Low-dose group	49	21 (42.86)	23 (46.94)	5 (10.20)	89.80%
Medium-dose group	49	24 (48.98)	16 (32.65)	9 (18.37)	81.63%
High-dose group	49	21 (42.86)	21 (42.86)	7 (14.29)	85.71%
*χ * ^2^					1.333
*P*					0.513

## Data Availability

The data used and/or analyzed during the current study are available from the corresponding author.
